The article "A Grounded Theory Construction of the eSports Endogenous Drive Model" was retracted in 2023. Reasons: signs of a paper mill; suspected computer-generated content; unreliable results or conclusions; lack of ethics approval or compliance.

# A Grounded Theory Construction of the eSports Endogenous Drive Model

**DOI:** 10.1155/2022/7731127

**Published:** 2022-09-30

**Authors:** Zhao Chen, Xiangui Bu

**Affiliations:** ^1^College of Physical Education, Zhengzhou University of Light Industry, Zhengzhou 450001, China; ^2^School of Competitive Sports, Shandong Sport University, Rizhao 276800, China

## Abstract

E-sports attracts a lot of time and energy from adolescents, making them happy to actively participate and even become addicted to the Internet. In order to reveal the mechanism of e-sports addiction and the mechanism of action, a model of e-sports internal drive was constructed by rooting qualitative analysis of interview data from 30 e-sports players, and the results of the study showed that the e-sports internal drive model consists of incentive setting (continuous incentive, variety of incentives, incentive can be redeemed, and incentive odds), task setting (can start over, flexible and free, can be completed, and specific goals), program setting (forming a team, simple interpersonal relationship, specific rules, timely feedback, fairness, simple operation, goal focus, quantified indicators, challenge difficulty, and training guidance), 3 dimensions, and 18 categories. The three dimensions are interrelated and synergistic eSports influencing factors. The establishment of this model enriches the relevant theories on the study of eSports endogamy and provides a reference basis for revealing the current social phenomenon of eSports game addiction among eSports players.

## 1. Introduction

E-sports is a sports competition in which video game competition reaches the level of “competition,” and as an emerging sports project, it has developed rapidly in recent years, and in 2017, the International Olympic Committee listed it as an official competition item of the 19th Asian Games. E-sports are based on e-games, information technology as a device, and confrontational e-competitions under unified competition rules, which have become a focus of attention and a phenomenon of society due to their novel form and attracting a large amount of youth time and energy [1]. One of the most important influences on the ability of e-sports to make adolescents happy to actively participate and even become addicted to the Internet is the internal drive of e-sports [2]. The design and experience of eSports can stimulate adolescents to awaken individual needs [3] and actively participate in eSports to meet individual needs, and the core logical mechanism and the mechanism of action are unclear. Currently, scholars at home and abroad study the types of attributes as well as mechanisms of eSports from different perspectives and levels and explore the pros and cons of eSports, but there is a relative lack of research on the factors influencing eSports endogamy, revealing that there is still a gap in the research on the internal mechanism of eSports players' addiction to the game. Therefore, this study has important theoretical and practical significance in constructing an endogenous model of eSports by adopting the research method of grounded theory.

The article "A Grounded Theory Construction of the eSports Endogenous Drive Model" was retracted in 2023. Reasons: signs of a paper mill; suspected computer-generated content; unreliable results or conclusions; lack of ethics approval or compliance.

## 2. Literature Review

E-sports players react differently to the same type of game because of the variability of individual e-sports players and the length of time they have been engaged in e-sports, which leads to differences in e-sports levels and can have different feeling experiences for the same video game [4]. By analyzing the types and tasks of eSports, it can be concluded that violent eSports will increase players' physically aggressive behavior and affect memory as well as cognition; violent eSports manifestations are mostly gun battles, swords, and physical fighting attacks; and wanting to win the game competition requires eSports players to conduct detailed research and repeated practice for the rules of the game, accumulate experience in the game, enhance the competitive proficiency, and, at the same time, will form conditioned reflexes [5, 6]. Heroic eSports tends to reduce players' radical thought behaviors, make players produce escape from the real world behavior, indulge in the virtual eSports world, manifest as negative work, unmotivated blood, obsessed with video games, and get pleasure and happiness experience in eSports so that their self-esteem is satisfied [7, 8]. E-sports players achieve self-actualization by gaining status and achievement in order to be recognized and paid attention to. The program motivation and partner recognition and their own happiness experienced by e-sports players in the process of participating in e-sports are lacking in the virtual world and satisfy the psychological needs of being needed and respected [9]; e-sports players are addicted to this unique psychological need space of e-sports, and thus, after being satisfied, role attachment arises, and after being recognized and needs are met virtually, eSports players become e-dependent [10]; the five properties of eSports characteristics such as interactivity, collaboration, equality, consumption, and addiction carry a strong goal orientation and can highlight self-worth in real games, so that the social interaction and psychological needs of eSports participants are doubly satisfied [11].

At present, scholars at home and abroad focus on the model design of eSports [4], eSports types [5], eSports task division [6], eSports role conversion [7], eSports process setting [8], eSports motivation [9], eSports psychology [10], and eSports characteristics [11]; and scholars at home and abroad are relatively scarce in their research on the internal drive of eSports and cannot internal mechanistic analysis of the phenomenon of eSports game addiction. This study analyzes the core influencing factors and internal logic of eSports endogenous drive by rooting in theoretical research methods, and on the basis of exploring the internal mechanism of eSports game addiction, in order to achieve positive guidance for youth to participate in eSports, this study has important theoretical and practical significance.

The article "A Grounded Theory Construction of the eSports Endogenous Drive Model" was retracted in 2023. Reasons: signs of a paper mill; suspected computer-generated content; unreliable results or conclusions; lack of ethics approval or compliance.

## 3. Research Methods

### 3.1. Literature Method

The literature search was conducted through China Knowledge Network, Wanfang Database, and International Journal Network, using “eSports,” “internal drive,” and “influencing factors” as keywords, and the research literature collected in the past 10 years (2012-2022) on the internal drive of e-sports at home and abroad was categorized and summarized to clarify the research lineage and the current situation of the research, which provided the basis of relevant literature for the study.

Woodworth first introduced the concept of endogenous drive in dynamic psychology: Columbia University Lectures, defining it as the internal motivation that drives individuals to satisfy their needs on the basis of needs [12]. Maslow defined it as the internal motivation that causes individuals to actively engage through external environmental stimuli [13]. Throughout the past decade of research, domestic and foreign scholars have generally emphasized the importance of the external environment as a trigger and the individual's motivation to awaken internal needs through external environmental stimuli, which in turn satisfies the individual's own needs [14]. The view that endogenous needs, through external stimuli, are carried out to motivate individuals to participate actively is in line with the mainstream psychological development [15]. This study considers eSports endogeneity as an influential factor in eSports stimulation to attract and drive individuals to actively participate in the eSports process.

### 3.2. Grounded Theory Research Method

Grounded theory as a qualitative research method complies with practice and provides a new methodological basis for eSports endogeneity research [16]. Unlike quantitative research methods that construct classes from hypotheses, the grounded theory research method instead enters the field, conducts field observation interviews, iteratively compares the collected data, extracts concepts and categories, identifies core categories and class relationships, and constructs theories from the bottom up [17, 18]. Since the theory of eSports endogamy is still in the exploration stage, no systematic analysis of eSports endogamy has been conducted in the previous research results, and therefore, quantitative research cannot be conducted. This study uses the grounded theory research method, which does not refer to existing theories, respects practice, and constructs a bottom-up model of eSports endogeneity according to the rooted research process.

The article "A Grounded Theory Construction of the eSports Endogenous Drive Model" was retracted in 2023. Reasons: signs of a paper mill; suspected computer-generated content; unreliable results or conclusions; lack of ethics approval or compliance.

Thirty eSports players who participated in the National eSports Open Finals in 2021 were selected as interviewees, and the interviewees were aged 18-37, with an average age of 25.53 years and an average of 6.97 years of gaming experience, with specific information on the interviewed information (see Table 1).

The first step was to enter the site for in-depth interviews and write memos to convert the interview data into textual texts [19]. The use of NVivo10 Chinese version of essential analysis software, which processes imported interview data, can effectively save the tediousness and workload of coding [20]. In the field of qualitative research, the use of data analysis software can effectively assist the researcher in completing coding and establishing categories and logical relationships [21]. Next, open coding was performed to extract the concepts and categories, then association coding was performed to determine the subordination, selection coding was performed to determine the core categories based on iterative comparison of relationships to complete the model construction, and finally mechanism analysis was performed to explore the logical mechanism and research findings of the model [22, 23]. Specific research procedures (see Figure 1).

Before the formal interviews, preinterviews were conducted. The purpose of the preinterview was to revise the semistructured interview outline, determine the focus and scope of the interview, revise the interview techniques and methods, and initially process the interview data. The content of the interviews revolved around the core questions: (1) what are the reasons why you like to play eSports? (2) What attracts you to eSports? (3) What aspects of eSports design make you feel awesome? (4) What factors of eSports can stimulate and drive you to participate in eSports? The interviewer controls the pace and orientation of the interview and quickly records new points that emerge during the interview so that follow-up questions can be asked to uncover more information. The interview time per person was 45-60 minutes. During the interview process for the same eSports experience and feelings, eSports players mostly have the same viewpoint. Through the pre-literature combing and pre-interview, the interviewees' representations were triangulated and inter-evaluated to enhance the objectivity of the interviewees' stated information.

The article "A Grounded Theory Construction of the eSports Endogenous Drive Model" was retracted in 2023. Reasons: signs of a paper mill; suspected computer-generated content; unreliable results or conclusions; lack of ethics approval or compliance.

## 4. Results and Analysis

Grounded theory is based on phenomena and practices and emphasizes the continuous interaction between information and analysis [24]. In this study, we strictly followed the Zagan coding process and coded the concepts and categories one by three levels, extracted them from the original interview data, and clustered them by repeatedly comparing their connotations and extensions and determining their subordination to obtain qualitative findings on the composition of core categories and relationships, so as to guarantee the reliability of the study [25].

Following the grounded theory research paradigm, the interview texts were openly coded word by word, sentence by sentence, and paragraph by paragraph, so that their concepts were naturally presented. The coding process maintained sensitivity to the theory, repeatedly comparing and deliberating the connotations and extensions of the concepts, and determining the subordination. After completing the open coding of 76,542 words of interview text and 8,643 words of memo, a total of 379 free tree nodes were obtained. After eliminating statements that were not related to the research topic, statements that appeared more than three times pointing to the same concept were selected and grouped and clustered into 46 concepts, and 18 categories were formed after repeated comparison of the concepts, which were sorted by the number of nodes that appeared as follows: continuous incentive, can be repeated, incentive diversity, incentive convertibility, incentive odds, flexibility and freedom, ability to complete, specific goals, forming a team, simple interpersonal relationships, specific rules, timely feedback, fairness, simple operation, goal focus, quantified indicators, challenge difficulty, and training guidance.

Secondary coding, i.e., associative coding was conducted on the basis of open coding to make connections between concepts and categories. 18 categories were established in open coding to compare and cluster the segmented concepts and categories to make the categories and dimensions specific. The comparison revealed the existence of three associative categories of task setting, procedure setting, and incentive setting (see Table 2).

Based on the correlation coding, the core category is formed to explore the causes of eSports endogenous drive. eSports task setting, program setting, and incentive setting are not isolated, but are interrelated and influential, and the three mechanisms work together to form the eSports endogenous drive setting, and the core category is identified as the eSports endogenous drive model, as shown in Figure 2.

The article "A Grounded Theory Construction of the eSports Endogenous Drive Model" was retracted in 2023. Reasons: signs of a paper mill; suspected computer-generated content; unreliable results or conclusions; lack of ethics approval or compliance.

E-sports players are driven by task-setting inducements, generate motivation and behavior, actively participate in the e-sports process, experience the e-sports program settings, get incentive setting stimulus in the process of completing the task goals, and this e-sports experience and incentive strengthens the e-sports behavior and promotes the next cycle to generate, so that e-sports players are more willing to invest in the e-sports process, forming a participation in e-sports closed loop. From the model, the three dimensions of incentive setting, program setting, and task setting synergistically influence the eSports internal drive.

From the correlational coding, it was found that the structure of the three dimensions, task setting, incentive setting, and program setting, was not equally important and had a primary and secondary importance. During the interviews and in the textual material, one or more of the main categories of incentive setting was mentioned more frequently than the other several times, proving that incentive setting is an important part of the eSports endogenous drive model. For the sake of research rigor, the statistical ranking of the three dimensions in the eSports internal drive model was conducted to evaluate the contribution value of each indicator by cardinality test. The frequency ranking of the first level dimensions revealed that motivation setting (180 frequencies, 36.73%), which accounted for the largest percentage, program setting (163 frequencies, 33.27%) was the second, and task setting (147 frequencies, 30.00%) was the smallest. The chi-square test showed a statistically significant distribution of differences in the three first-level dimensions (*X*^2^ = 61.396, *p* ≤ 0.001) (see Table 3).

The analysis of the frequency of the secondary dimensions of the eSports internal drive model shows (see Table 4) that continuous motivation and being able to start over are the most mentioned categories by the interviewers, training guidance is mentioned the least, and since the interviews are all senior players, less attention is paid to the guidance of junior eSports.

Most of the factors of internal drive influence factors can find corresponding support in previous studies, as shown in Table 5. Task setting dimension, eSports endogenous drive influence factors specific goal, able to complete, can be repeated, and flexible and free found validation in the previous literature.

Among the incentive setting dimensions, previous studies have mostly focused on continuous incentive, incentive diversity among eSports internal drive influencing factors, while ignoring incentive odds, incentive convertibility, which is a new finding of this paper. Program setting dimension, timely feedback, simple interpersonal relationship, and training guidance did not find verification, which belongs to the innovation proposed in this paper. Previous studies focused on challenge difficulty, rule specificity, team formation, goal focus, target quantification, and operational simplicity of eSports internal drive influencing factors, ignoring the three influencing factors of timely feedback, simple interpersonal relationship, and training guidance, which is a new finding of this paper. This study for the first time constructs a model of eSports internal drive by 3 dimensions of task setting, incentive setting, and procedure setting, with 18 categories interrelated, which is a breakthrough of the previous research results. By comparing the 3-dimensional and 18 main categories of eSports internal motivation model constructed by the three-level coding with the previous studies, we found that the previous studies focused on game design, game operation, game effectiveness, etc. and failed to systematically determine the relationship and logical mechanism of each influencing factor, and the studies were relatively isolated and scattered. The bottom-up model of eSports in this study covers some of the influencing factors ignored by previous studies and clusters out the logical relationships among the influencing factors as a whole, which is more systematic and comprehensive compared with the previous studies. Therefore, the eSports endogeneity model constructed in this study can better explain the influence mechanism of eSports endogeneity than previous theories.

The article "A Grounded Theory Construction of the eSports Endogenous Drive Model" was retracted in 2023. Reasons: signs of a paper mill; suspected computer-generated content; unreliable results or conclusions; lack of ethics approval or compliance.

## 5. Discussion

Incentive setting is to stimulate e-sports players and set incentives, for attracting players to participate in e-sports has an important role in the guidance, from the novice field to the master field of e-sports process, e-sports from simple to complex, increasing the difficulty coefficient, but each level set incentives measures to effectively improve the motivation of players, their continuous promotion, to achieve a sense of self-worth identity, increased willingness to participate. In the process of continuous advancement, players achieve a sense of self-worth and increase their willingness to participate. The 180 tree nodes about incentive setting are found from the open code and associated code, which is the highest percentage among the three dimensions. In the incentive setting, it is further divided into four parts: continuous incentive, incentive diversity, incentive convertibility, and incentive chance.

Continuous incentive accounts for 58 reference points, accounting for 32%, which shows that continuous incentive accounts for the largest proportion in eSports incentive settings and is the most attractive to eSports players. Most of the eSports players in the interview mentioned that the continuous game rewards can make players have higher participation enthusiasm in the game. The diversity of incentive accounts for 45 reference points, accounting for 25%, each level in e-sports rewards is different, there are points, equipment, weapons, life value, etc. It is because of the diversity of e-sports incentives to make players happy to explore to find new tasks, complete new tasks, so as to get different e-sports rewards. Incentive redeemable account for 40 reference points, accounting for 22%, players in the eSports process to complete each level of the task will be different rewards, when the reward amount reaches a certain contribution value can be exchanged and traded, you can buy more advanced equipment and weapons, you can also give equipment to other players to trade, in exchange for contribution value and points. Incentive odds accounted for 38 reference points, accounting for 21% of the total. In different stages of a mission or a level, some rewards are probabilistic, and it is these uncertainties that increase the fun and involvement of the game, making eSports players match their personal needs and thus balance the game process.

Task setting refers to the means of measures taken by eSports in setting goals in order to keep the game players highly enthusiastic and engaged. The 147 tree nodes occupied by task setting include four parts: can be repeated, flexible and free, can be completed, and specific goals. Can start over accounted for 46 reference points, or 31% of the total. After losing in eSports due to mistakes or inferior skills to their opponents, players can start the game again and continue the task, so that they have no worries and can experience the game with a peaceful mind. The reason is that from beginners to advanced players, they need to keep repeating and replaying, accumulating experience and skills, mastering the rules of the game, and improving their game level. Flexibility and freedom account for 37 reference points, accounting for 25%. Players in e-sports can freely choose characters and scenes and can freely team up to compete, reducing the fetters and constraints, and not being overly set up to sway and restrict, which is also esteemed by e-sports players.

Being able to complete accounts for 34 reference points, accounting for 23%. In the eSports task set, after repeated practice and try each level of the task can be completed, but also to attract players repeatedly failed important reason. The sense of accomplishment of completing each level of the task in the participation experience eSports also stimulates eSports participants. The goal specifically accounts for 30 reference points, accounting for 20%, in each eSports situation and level, what needs to be defeated or built has clear requirements, players complete each task according to specific goals and then pass the level, into the higher levels, and the points earned to participate in the entire eSports ranking, according to different regions to show the number of provincial and urban rankings, directly stimulate the eSports players sense of participation.

The article "A Grounded Theory Construction of the eSports Endogenous Drive Model" was retracted in 2023. Reasons: signs of a paper mill; suspected computer-generated content; unreliable results or conclusions; lack of ethics approval or compliance.

Program setting is the program setting for eSports players to get a good experience in the game process. The 163 tree nodes in the program setting include ten parts of forming a team, simple interpersonal relationship, specific rules, timely feedback, fairness, simple operation, goal focus, quantified indicators, challenge difficulty, and training guidance. Forming a team accounted for 27 reference points, accounting for 17%, and most players in the interviews mentioned that forming a team to fight is their preferred way of eSports, both for solo eSports and for team participation in eSports, both of which can be ranked in points, and teamwork and formation also improve the participation of eSports players. Interpersonal relationship simple accounted for 24 reference points, accounting for 15%, e-sports players in the game process only need to complete the corresponding tasks, in the team process into also collaborate to complete each level of the task, communication is simple, the interview players basically a sentence can understand what they do, there is no other too much communication, the technical level of the division of labor is more simple and direct, easy to accept the implementation. Rules specific account for 18 reference points, accounting for 11%, in the eSports each level set, what weapons and equipment to use, how to score and complete the task rules are clear and specific, players only need to follow the eSports rules in a sequential manner. Feedback timely and fair each accounted for 17 and 16 reference points, the proportion is basically the same, because in eSports can be found in a timely manner life value, blood value, and score in order to feedback to the player to take measures and methods to complete the task, while the rules are unified, so fair is the eSports guidelines that players are agreed. Simple operation and target focus each account for 15 and 14 reference points, the proportion is basically the same. Players in e-sports only need to simply operate the keyboard or cell phone, and each level task is more focused, players only need to complete the task to pass the level, and in the interview, most players think that e-sports take up a lot of time because the attention is focused on each level task.

The article "A Grounded Theory Construction of the eSports Endogenous Drive Model" was retracted in 2023. Reasons: signs of a paper mill; suspected computer-generated content; unreliable results or conclusions; lack of ethics approval or compliance.

Indicators can be quantified accounted for 13 reference points, accounting for 8%, e-sports players can clearly know the game process and the current state are an important factor to let e-sports go on, and players can use their own wisdom to constantly adjust the e-sports path and optimization methods. Challenge difficulty and training guidance accounted for 10 and 9 reference points, respectively, and the proportions were basically the same. E-sports players in the process of advancement in the competitive difficulty is increasing, its order to reflect their own ability and value achievement will continue to upgrade the ranking, while the e-sports itself will prompt to note and complete the task guidance, can make the e-sports players in the tips, and help for the game cycle participation.

## 6. Conclusion

By constructing the eSports internal drive model by open coding, associative coding, and selective coding, it is proposed that the eSports internal drive model is a three-dimensional integrated model consisting of three dimensions: incentive setting, task setting, and program setting. The 18 categories of eSports internal drive are continuous motivation, replayable, incentive diversity, incentive convertibility, incentive odds, flexible and free, able to complete, specific goal, forming a team, simple interpersonal relationship, specific rules, timely feedback, fairness, simple operation, goal focus, quantified target, challenge difficulty, and training guidance. The 18 categories were grouped into three dimensions: incentive setting, task setting, and procedure setting through open coding and correlation coding. The incentive setting dimension includes four categories: continuous incentive, incentive diversity, incentive redeemable, and incentive odds. The task setting dimension consists of four categories: repeatable, flexible and free, capable of completion, and specific goals. The procedure setting dimension includes ten categories consisting of forming a team, simple interpersonal relationship, specific rules, timely feedback, fairness, simple operation, goal focus, quantified targets, challenge difficulty, and training guidance.

The model of eSports endogenous drive constructed based on Grounded theory systematically analyzes the influencing factors of eSports endogenous drive, which is a breakthrough to the previous research results and helps to reveal the internal mechanism of the current social phenomenon of gaming addiction among eSports players and provides a relevant theoretical foundation for the empirical study of eSports endogenous drive. The construction of the eSports internal drive model based on the grounded theory can help explain the social phenomenon of eSports game addiction. In the future, through the eSports internal drive assessment scale, empirical research can be conducted on the eSports game addiction group to decipher the internal mechanism of game addiction, so as to make targeted interventions for this group.

The article "A Grounded Theory Construction of the eSports Endogenous Drive Model" was retracted in 2023. Reasons: signs of a paper mill; suspected computer-generated content; unreliable results or conclusions; lack of ethics approval or compliance.

## Figures and Tables

**Figure 1:** Procedure chart of grounded theory research.

**Figure 2:** eSports internal drive model.

**Table 1:** List of basic information of the interviewees.

Number	Age	Game years	Career	Number	Age	Game years	Career
001	19	5	College students	016	30	10	Property manager
002	25	7	Nurse	017	24	6	Freelance
003	33	9	Elementary school teachers	018	27	8	Electrician
004	28	6	Engineer	019	29	8	Doctors
005	18	4	College students	020	18	4	College students
006	20	5	Company security	021	23	5	Corporate finance
007	26	7	E-commerce	022	35	11	University faculty
008	33	10	Individual owners	023	24	6	Baker
009	21	6	Company cashier	024	32	9	Company manager
010	18	4	Technical school students	025	19	5	Factory security
011	20	5	Company staff	026	27	7	Electric welding technician
012	30	7	Secondary school teachers	027	37	13	University faculty
013	34	9	Individual owners	028	29	9	Individual owners
014	21	7	Sales staff	029	22	5	Property finance
015	19	5	Sales staff	030	25	7	Doctors

**Table 2:** Demonstration of the results of the eSports endogamy association coding: concepts and categories.

Associative coding (reference points)	Open coding (reference points)	Original statement enumeration
Incentive settings (180)	Continuous motivation (57) Chance of motivation (38) Diversity of motivation (45) Incentive redeemable (40)	Players will be rewarded for each task they complete; the rewarded equipment appears randomly, with weapons and clothes; their own equipment can be exchanged with other players or sold.

Program settings (163)	Challenge difficulty (10) Rules specific (18) Forming a team (27) Fairness (16) Target focus (14) Timely feedback (17) Quantification of indicators (13) Simple interpersonal relationships (24) Training guidance (9) Easy to operate (15)	The higher the number of levels you play, the more accomplished you are; which level has double points are relatively clear; find a high level team win rate is mostly; everyone in the game is the same; what specific tasks to do are very clear; from the blood bar display to know their life value; kill a monster experience value plus three hundred; we just need to play the game together; each level has instructions; point a keyboard or cell phone page can be operated.

Task settings (147)	Goal specific (30) Able to complete (34) Can start over (46) Flexibility and freedom (37)	The level specifies the task of each level; anyway, it can be completed; if you cannot beat it and die, you can start over; there are a dozen tasks each day that you can choose at will according to your own expertise.

The article "A Grounded Theory Construction of the eSports Endogenous Drive Model" was retracted in 2023. Reasons: signs of a paper mill; suspected computer-generated content; unreliable results or conclusions; lack of ethics approval or compliance.

**Table 3:** Ranking the importance of internal drive level 1 dimensions.

Level 1 dimension	Sort by	Frequency	%	*X* ^2^	*p*
Incentive settings	1	180	36.73		
Program settings	2	163	33.27	61.396	≤0.001
Task settings	3	147	30.00		

**Table 4:** Ranking the importance of the second-level dimensions of internal motivation.

Level 1 dimension	Secondary dimension	Frequency	%	Sort by
Incentive settings	Continuous motivation	57	11.63	1
	Incentive odds	38	7.76	5
	Diversity of motivation	45	9.18	3
	Incentive redeemable	40	8.16	4

Program settings	Challenge difficulty	10	2.04	17
	Rules specific	18	3.67	11
	Forming a team	27	5.10	9
	Fairness	16	3.26	13
	Target focus	14	2.86	15
	Timely feedback	17	3.47	12
	Quantification of indicators	13	2.65	16
	Simple interpersonal relationships	24	4.90	10
	Training guidance	9	1.84	18
	Easy to operate	15	3.06	14

Task settings	Specific objectives	30	6.12	8
	Able to complete	34	6.94	7
	Can start over	46	9.39	2
	Flexibility and freedom	37	7.55	6

**Table 5:** Validation of the theoretical categories by comparison of related literature.

Number	Category	Comparative examples of representative literature	Number	Category	Comparative examples of representative literature
1	Specific objectives	Shute V [2]	10	Fairness	Ma Xiaoqiang [10]
2	Able to complete	Shute V [2]	11	Target focus	Bailey, West [5],
3	Can start over	Bailey, West [4],	12	Quantification of indicators	Anderson [4]
4	Flexibility and freedom	Anderson [3]	13	Easy to operate	Feng Gang [8]
5	Continuous motivation	Sestir, M. A [5].	14	Incentive odds	The discovery of the quality of this article
6	Motivating diversity	Sestir, M. A [5].	15	Incentive redeemable	The discovery of the quality of this article
7	Challenge difficulty	Wei Hua [8]	16	Timely feedback	The discovery of the quality of this article
8	Rules specific	Rooji et al. [6]	17	Simple interpersonal relationships	The discovery of the quality of this article
9	Forming a team	Ma Xiaoqiang [9]	18	Training guidance	The discovery of the quality of this article

## Data Availability

All the data for this study is to be accessed by request.
